# Prognostic Value of Lactate Dehydrogenase, Melanoma Inhibitory Protein, and S-100B Protein in Patients with Malignant Melanoma

**DOI:** 10.1155/2022/9086540

**Published:** 2022-10-04

**Authors:** Shuwen Fan, Xiao Liu, Yizhu Wu, Ke Li, Xiaoyu Zhao, Wei Lin, Jianjiang Liu

**Affiliations:** Department of Burn and Plastic Surgery, The First Affiliated Hospital of Soochow University, Suzhou, Jiangsu 215000, China

## Abstract

**Objective:**

This investigation probed the prognostic potential for lactate dehydrogenase (LDH), melanoma inhibitory activity protein (MIA), and S-100B protein in cases of malignant melanoma.

**Methods:**

84 cases were segregated into effective cohort (*n* = 64) and ineffective cohort (*n* = 20) depending on clinical efficacy. The cases were followed up for three years and segregated into mortality cohort (*n* = 29) and survival cohort (*n* = 55) depending upon 3-year survival. Serum LDH, MIA, and S-100B levels were compared across the effective and ineffective cohorts. Serum LDH, MIA, and S-100B levels in cases of different clinical stages were comparatively analyzed, with correlations of these indicators with the clinical stage being evaluated. ROC evaluated the prognostic potential of serum LDH, MIA, and S-100B. Cases were segregated into the high-level and low-level cohorts according to serum LDH, MIA, and S-100B levels, and the survival rates of cases were compared.

**Results:**

The levels of LDH, MIA, and S-100B in the effective cohort were significantly lower than those in the ineffective cohort. The AUC value of the composite indicator of serum LDH, MIA, and S-100B for effectiveness evaluation was (0.839). Serum LDH, MIA, and S-100B levels were positively linked to the clinical stage. AUC value of the composite indicator of serum LDH, MIA, and S-100B for prognosis evaluation prediction (0.942) was elevated compared to LDH (0.632), MIA (0.732), or S-100B (0.828) alone. Survival rate of cases of LDH ≥30.56 mg/L (57.14%, 32/56) was lower than that of cases of LDH <30.56 mg/L (82.14%, 23/28) (log-rank χ^*2*^ = 4.672, *P* < 0.05). The survival rate of MIA ≥5.34 ng/mL cases was lower than that of MIA <5.34 ng/mL cases. The survival rate of cases of S-100B ≥ 1.03ug/L was lower than that of S-100B < 1.03ug/L.

**Conclusion:**

Serum LDH, MIA, and S-100B protein levels are linked to the clinical stage. The lactate dehydrogenase, melanoma inhibitory protein, and S-100B protein are of good clinical effectiveness and have the prognostic potential for cases of malignant melanoma.

## 1. Introduction

Malignant melanoma (MM) is a malignant tumor of epithelial origin, and its incidence has shown an increasing trend in recent years. Ultraviolet radiation (UV) and malignant changes in moles are risk factors for MM. Surgical resection, radiotherapy, and chemotherapy are often employed in the clinical treatment of melanoma. It is reported that the 5-year survival rate of cases of MM in the United States is 98%, and the 5-year survival rate in cases of stage IV melanoma is 3%. Therefore, early prediction of melanoma cases is crucial, which is conducive to the personalized and accurate treatment of cases of MM [1–3].

Serum-based lactate dehydrogenase (LDH) is a critical member of the glycolytic enzymatic family, which might mediate the oxidation of lactic acid to pyruvate and increase serum LDH levels. Emerging evidence indicates that LDH is associated with heavy tumor load and poor prognosis [4, 5]. Melanoma inhibitory activity protein (MIA) is closely related to malignant tumor proliferation, metastasis, and invasion. Moreover, MIA could accelerate tumor cell apoptosis and block tumor angiogenesis [6, 7]. MIA can specifically inhibit the adhesion of melanoma cells to fibronectin and laminin, affecting tumor cell metastases; S-100b protein is highly expressed in MM and is also found to be elevated in the normal population [8–10]. S-100B proteomic expression can reflect the tumor load of cases and is related to the recurrence and progression of the disease.

The current study explores the predictive value of LDH, MIA, and S-100B protein levels in the prognosis of patients with malignant melanoma.

## 2. Material and Methods

### 2.1. General Data

Eighty-four cases of advanced melanoma treated in our hospital from January 2013 to February 2019 were accepted, including 53 males and 31 females. Age ranged from 41 to 72 years, with a mean of 55.65 ± 5.72 years. The Hospital Ethics Committee accepted this investigation. Inclusion criteria: (1) All subjects were in line with the relevant standards of *Clinical Practice Guidelines for Pathological Diagnosis of Melanoma (2021 edition)* [11]; (2) All cases were the first onset; (3) All subjects had an expected survival time >3 months; (4) All subjects had complete clinicopathological data; (5) All subjects volunteered to participate in this study. Exclusion criteria: (1) Cases aged >75 years; (2) Cases of other malignant tumor diseases; (3) No drug, laser, or radiotherapy was given before enrollment; (4) Cases of autoimmune diseases; (5) Cases of severe cardiac/hepatic/renal dysfunction; (6) Cases of distant metastasis; (7) Cases of severe adverse reactions to chemotherapy.

### 2.2. Therapeutic Methods

After admission, all patients received relevant examination and chemotherapy risk assessment and were treated with high-dose recombinant human *α*-2b interferon combined with conventional chemotherapy. The recombinant human interferon *α*-2b of 3 million *U* + injection 2 mL was injected subcutaneously on *d* 3, 6 million *U* + 2 mL on *d* 6 and 9 million *U* + 2 mL on *d* 9. The treatment lasted 4 courses, 21 days as the course of treatment. The conventional chemotherapy regimen was dacarbazine + cisplatin + vincristine + doxorubicin, and the administration standard was as follows: intravenous drip of dacarbazine 100 mg/m^2^ during d1 to d5; cisplatin 20 mg/m^2^, vincristine 2 mg, and doxorubicin 50 mg were given intravenously during d1 to d8. On d1, 80 mg/m^2^ of lomustine was taken orally. The treatment continued for four courses with 21 days as a course.

### 2.3. Clinical Effectiveness Evaluation

All cases were assessed depending on effectiveness parameters for solid tumors [12] and were segregated into complete response (CR), partial response (PR), stable disease (SD), and progressive disease (PD). CR: tumor diameter was reduced by ≥ 80%, no new lesions were developed, and the response was maintained for at least four weeks; PR: the tumor diameter was reduced by 50% to 79%, and the response remained for at least four weeks; SD: the tumor diameter was reduced by 30%∼49%; PD: the tumor diameter was reduced by <29% or a had an increase, or new lesions emerged. Total response = CR + PR + SD.

### 2.4. Prognostic Evaluation

All cases were followed up remotely/outpatient-based follow-up for three years. Cases were segregated into mortality cohort and survival cohort according to 3-year survival.

### 2.5. Detection of Serum LDH, MIA, and S-100B Protein Levels

10 mL of fasting venous blood was taken from individual cases in the morning and centrifuged at 2500 r/min for 15 min. The upper serum was collected and stored at −80°C. Serum LDH, MIA, and S-100B proteomic expression were identified through enzyme-linked immunosorbent assay (ELISA). The normal value of serum LDH is 100–300u/l. The average level of serum S-100B > 0.4 *μ*g/kg indicates a poor prognosis.

### 2.6. Observation Indicators

(1) Serum LDH, MIA, and Smur100 B levels were compared between valid and ineffective cohorts. (2) The clinical value of serum lactate dehydrogenase, lactam, and Smur100B levels was evaluated by ROC curve. (3) Serum LDH, MIA, and S-100B levels in cases of different clinical stages were compared to evaluate the correlation of serum LDH, MIA, and S-100B levels with clinical stages. (4) The levels of serum lactate dehydrogenase, lactam, and Smur100B, including survival time and mortality cohort, were compared. (5) The prognostic potential of serum lactate dehydrogenase, lactam and Smur100 B levels were evaluated by ROC. (6) According to serum LDH, MIA, and S-100B levels, cases were segregated into the high-level and low-level cohorts. The survival curves of cases of differing serum LDH, MIA, and S-100B levels were evaluated, and the survival rates of cases of different levels were compared.

### 2.7. Statistical Analysis

Data were processed through SPSS® 24.0 and GraphPad Prism 5. Descriptive statistics were expressed as Mean ± SD ($\bar{x}$ ± S). Categorical variables were represented as *n* and %, chi-square test was employed to analyze the across cohorts, and rank sum test was employed for ranked data. The prognostic values of lactate dehydrogenase, melanoma inhibitory protein, and S-100B protein in patients with malignant melanoma in different groups were calculated by the Kaplan–Meier method, and the cumulative incidence was compared between groups by the log-rank method. ROC curve was employed to assess the evaluation value of serum LDH, MIA, and S-100B levels for the clinical effectiveness in patients with MM. Spearman correlation analysis was employed to evaluate the correlation across the AJCC stage and serum LDH, MIA, and S-100B levels. Log-rank χ^*2*^ test was employed to evaluate the survival rate among the two cohorts. All tests were two-sided, and *P* < 0.05 was considered a statistical significance.

## 3. Results

### 3.1. Clinical Effectiveness

A total of 11 cases of CR, 28 cases of PR, 25 cases of SD, and 20 cases of PD were identified. The total effective rate was 76.19% (64/84).

### 3.2. Comparison of Serum LDH, MIA, and S-100B Levels between the Influential and Ineffective Cohort

Serum LDH, MIA, and S-100B levels in the influential cohort were reduced compared with those in the ineffective cohort (all *P* < 0.05, Table 1).

### 3.3. Association between Serum LDH, MIA, and S-100B Levels and Clinical Effectiveness

The AUC value of the combined evaluation with serum LDH, MIA, and S-100B (0.839) was elevated compared to LDH alone (0.699) (*P* < 0.05, Table 2 and Figure 1).

### 3.4. Comparative Analysis of Serum LDH, MIA, and S-100B Levels in Differing Clinical Stages

Serum LDH, MIA, and S-100B levels in stages II, III, and IV were elevated compared with those in stage I, the levels of the above indicators in stage III and IV were elevated compared with those in stage II, and the levels in stage IV were elevated compared with those in stage III (all *P* < 0.05, Table 3).

### 3.5. Correlation Analysis of Serum LDH, MIA, And S-100B Levels with Clinical Stage

Serum LDH, MIA, and S-100B levels were positively linked to the clinical stage (all *P* < 0.05, Figure 2).

### 3.6. Comparative Analysis of Serum LDH, MIA, and S-100B Levels across Survival Cohort and Mortality Cohort

The serum LDH, MIA, and S-100B levels in the survival cohort were reduced compared with those in the mortality cohort (all *P* < 0.05, Table 4).

### 3.7. Prognostic Value of Serum LDH, MIA, and S-100B Levels

The AUC value of the combination of serum LDH, MIA, and S-100B indicators to predict prognosis (0.942) was better than LDH (0.632), MIA (0.732), or S-100B (0.828) alone (all *P* < 0.05, Table 5 and Figure 3).

### 3.8. Survival Curve Analysis of Cases of Differing Serum LDH, MIA, and S-100B Levels

The survival rate of cases of LDH ≥30.56 mg/L (57.14%, 32/56) was lower than that of cases of LDH<30.56 mg/L (82.14%, 23/28) (log-rank k χ^*2*^ = 4.672, *P* < 0.05). The survival rate of cases of MIA ≥5.34 ng/mL (55.38%, 36/65) was lower than that of cases of MIA <5.34 ng/mL (100%, 19/19) (log-rank χ^*2*^ = 10.810, *P* < 0.05). The survival rate of cases of S-100B ≥ 1.03 ug/L (26.77%, 17/40) was lower than that of cases of S-100B < 1.03 ug/L (86.36%, 38/44) (log-rank χ^*2*^ = 17.060, *P* < 0.05) (Figure 4).

## 4. Discussion

Cutaneous melanoma is a highly malignant tumor with a high recurrence rate and uncomplicated metastasis. Its prognosis is related to many factors, such as treatment timing, treatment method, and the presence of metastasis. Surgical resection is the first choice for clinical treatment of MM, but due to the number of lesions, anatomical location, and recurrence after surgical resection, surgery is not suitable for all cases of MM. Immunotherapy, targeted therapy, and other methods have been gradually applied to MM treatment. Recombinant human *α*-2b interferon is a secretory protein with antitumor, antivirus, and immunomodulatory functions. By imitating the function of interferon in the body, it plays a variety of biological activities, has the advantage of a fast metabolism, and can reduce the burden on the liver. In the present study, recombinant human interferon *α*-2b showed an excellent effect in MM treatment, with a total effective rate of 76.19% (64/84).

LDH exists widely in many human tissues and is involved in the glycolysis pathway. It is reported that glycolysis and LDH activity in malignant tumors is significantly higher than that in normal tissues. Therefore, the serum lactate dehydrogenase level in cancer patients increases, and lactate dehydrogenase is related to the prognosis of various malignant tumors [13, 14]. Previous studies have shown that LDH is an independent risk factor for prognosis MM cases, and the serum LDH level in MM cases is high [15, 16]. In addition, it has been reported that serum LDH levels have shown varying degrees of elevation, indicating anaerobic glycolysis in tissues before imaging manifestations in tumor cases. MIA is a secretory tumor growth suppressor that can regulate cell adhesion by specifically inhibiting melanoma cell adhesion to fibronectin laminin to regulate melanoma cell shedding from the extracellular matrix and ultimately affect tumor metastases. Evidence has indicated that MIA was highly expressed in the serum of MM patients, while overexpression of MIA may indicate a poor prognosis [17, 18]. S-100b protein is an acidic calcium-binding protein, widely existing in normal tissue cells of nerve ectodermal leaf, mesoderm, and ectoderm, or originating from cell tumors.

Most of them exist in cells and can be released into the blood when cells proliferate massively. It has been reported that S-100B protein is rarely expressed in nonmelanocyte tumors, and serum S-100B protein level is intimately linked with individual case tumor load. In addition, serum S-100B protein can reflect the therapeutic effect of patients and be employed as a prognostic indicator of MM. The elevation of the S-100B protein level in serum of MM cases occurred earlier than the onset of clinical symptoms [18, 19]. In the present study, the serum LDH, MIA, and S-100B levels in the influential cohort were reduced compared to the ineffective cohort, and the AUC value of the combined evaluation for clinical effectiveness with serum LDH, MIA, and S-100B (0.839) was higher than that with LDH (0.699) alone (*P* < 0.05). The result indicated that serum LDH, MIA, and S-100B levels are related to the therapeutic effect of recombinant human *α*-2b interferon on MM. These indicators can be employed to predict the clinical effectiveness of recombinant human *α*-2b interferon on MM.

AJCC stage is a commonly employed tool for clinically evaluating the severity and prognosis of malignant tumor diseases. However, the clinical application is subject to the subjective influence of the operator, which cannot be objective and cannot be applied to ultra-early diagnosis. In the present study, serum LDH, MIA, and S-100B levels of AJCC stage II, III, and IV were higher than those of stage I, serum LDH, those of stage III and IV were higher than those of stage II, those of stage IV were higher than those of stage III, suggesting the correlation of serum LDH, MIA, and S-100B levels with AJCC tumor stage. Spearman correlation analysis showed that serum LDH, MIA, and S-100B levels were positively linked to the clinical stage (all *P* < 0.05), suggesting that the elevation of serum LDH, MIA, and S-100B may be related to tumor progression. Detecting these tumor markers is convenient and plays a particular role in predicting recurrence and metastasis. Serum LDH, MIA, and S-100B levels are positively linked to the clinical stage, so the stability or progression of the disease can be judged based on the changes in serum LDH, MIA, and S-100B levels.

Tumor cell metabolism is unique and characterized by increased glucose uptake and glycolysis. Tumor cells metabolize energy through glycolysis regardless of oxygen availability. LDH is a crucial catalytic enzyme in the glycolysis pathway. LDH can promote pyruvate to generate lactate, and lactate accumulation can provide an acidic microenvironment conducive to tumor growth, invasion, and metastasis [20, 21]. Previous studies have shown that MIA and S-100B are closely related to the occurrence and development of MM [22, 23]. In the present study, the levels of serum LDH, MIA, and S-100B in the survival cohort were significantly reduced compared to those in the mortality cohort (all *P* < 0.05); the AUC value of serum LDH, MIA, and S-100B combined indicator (0.942) was higher than that with LDH (0.632), MIA (0.732), or S-100B (0.828) alone (all *P* < 0.05); the survival rates of cases of LDH ≥30.56 mg/L, MIA ≥5.34 ng/mL, or S-100B ≥ 1.03ug/L were lower than those of cases of LDH <30.56 mg/L, MIA ng/mL < 5.34, or S-100B < 1.03 ug/L. All these results suggested that serum LDH, MIA, or S-100B levels can be employed to evaluate the prognosis of MM. Elevated LDH levels are associated with the glycolysis pathway, which provides a favorable environment for tumor growth. MIA explicitly inhibits the adhesion of melanoma cells to fibronectin and laminin, affecting the metastasis of tumor cells, and its specific mechanism remains to be further explored. Previous studies have shown that S-100B is positively linked to the MM stage [24, 25], which is consistent with the results of the present study.

To sum up, serum LDH, MIA, and Smur100 B levels correlate with the clinical stage, and their combined detection is of value in evaluating the therapeutic effect and predicting the prognosis of MM cases. The limitation of this study is that a single-center retrospective study may lead to statistical bias. In a further study, a multicenter analysis could be performed to assess the correlation between serum lactate dehydrogenase, lactam, and Smur100B levels and MM.

## Figures and Tables

**Figure 1:** ROC curve analysis of evaluation value of LDH, MIA, and S-100B levels for clinical effectiveness. Note: Compared with combination, ^*∗*^*P* < 0.05.

**Figure 2:** Correlation analysis of serum LDH, MIA, and S-100B levels with clinical stage.

**Figure 3:** Prognostic value of serum LDH, MIA, and S-100B levels. Note: Compared with combination, ^*∗*^*P* < 0.05.

**Figure 4:** Survival curve analysis of cases of differing serum LDH, MIA, and S-100B levels.

**Table 1:** Comparison of serum LDH, MIA, and S-100B levels between the two cohorts ($\bar{x}$ ± *s*).

Cohort	LDH (mg/l)	MIA (ng/ml)	S-100B (ug/l)
Effective cohort (*n* = 64)	37.84 ± 16.35	7.68 ± 4.10	1.03 ± 0.45
Ineffective cohort (*n* = 20)	51.62 ± 20.44	13.11 ± 4.63	1.71 ± 0.68
*t*-value	3.095	5.019	4.177
*P*-value	0.003	<0.001	<0.001

**Table 2:** Evaluation value of serum LDH, MIA, and S-100B levels for clinical effectiveness.

Indicator	Cut-off value	AUC	SE	95% CI
LDH	31.56	0.699^*∗*^	0.064	0.573∼0.825
MIA	11.73	0.789	0.058	0.686∼0.911
NWR	1.27	0.794	0.059	0.678∼0.909
Combination		0.839	0.053	0.735∼0.943

**Table 3:** Comparative analysis of serum LDH, MIA, and S-100B levels in differing clinical stages (*x* ± *s*).

AJCC stage	LDH (mg/l)	MIA (ng/ml)	S-100B (ug/l)
Stage I (*n* = 9)	15.63 ± 1.89	2.99 ± 1.48	0.47 ± 0.17
Stage II (*n* = 38)	30.19 ± 4.31^a^	6.39 ± 2.75^a^	0.97 ± 0.37^a^
Stage III (*n* = 24)	51.53 ± 5.43^ab^	11.58 ± 2.70^ab^	1.34 ± 0.42^ab^
Stage IV (*n* = 13)	71.52 ± 10.28^abc^	15.84 ± 2.83^abc^	2.06 ± 0.47^abc^
*F*-value	250.393	64.176	37.142
*P*-value	<0.001	<0.001	<0.001

Note: Compared with stage I, ^a^*P* < 0.05; compared with stage, ^b^*P* < 0.05; Compared with stage III, ^c^*P* < 0.05.

**Table 4:** Comparative analysis of serum LDH, MIA, and S-100B levels across survival cohort and mortality cohort ($\bar{x}$ ± *s*).

Cohort	LDH (mg/l)	MIA (ng/ml)	S-100B (ug/l)
Survival cohort (*n* = 55)	37.97 ± 16.41	7.62 ± 4.38	0.96 ± 0.42
Mortality cohort (*n* = 29)	47.10 ± 20.31	11.54 ± 4.58	1.62 ± 0.62
t-value	2.230	3.840	5.087
*P*-value	0.029	<0.001	<0.001

**Table 5:** Prognostic values of serum LDH, MIA, and S-100B levels.

Indicator	Cut-off value	AUC	SE	95% CI
LDH	30.56	0.632^*∗*^	0.063	0.509∼0.755
MIA	5.34	0.732^*∗*^	0.055	0.625∼0.839
S-100B	1.03	0.828^*∗*^	0.044	0.742∼0.913
Combination		0.942	0.028	0.888∼0.997

## Data Availability

The labeled dataset used to support the findings of this study are available from the corresponding author upon request.
